# A Product Styling Design Evaluation Method Based on Multilayer Perceptron Genetic Algorithm Neural Network Algorithm

**DOI:** 10.1155/2021/2861292

**Published:** 2021-12-02

**Authors:** Jie Wu

**Affiliations:** School of Anyang Institute of Technology, Anyang, Henan 45500, China

## Abstract

Products no longer exist simply as carriers of useful functions, but more and more consumers are beginning to pay attention to the spiritual aspects of the feelings brought by products. This paper brings machine learning algorithms to the discipline of industrial design and proposes a method to evaluate the design of product shapes using a multilayer perceptron genetic algorithm neural network (GA-MLP-NN) algorithm, quantifying the product shape, using computer-aided design technology to achieve shape optimization, shape, and color scheme generation, and using interactive feedback with users to finally generate a product shape with market demand. In this paper, we use the combinatorial innovation method to arrange and combine the detail elements in the solution library to generate the modeling solution, combine the multilayer perceptron genetic algorithm neural network algorithm with product modeling, and establish the interactive genetic modeling system for the product, use this system to design the product modeling solution, and finally get the product modeling solution satisfied by the target users; using the multilayer perceptron genetic algorithm neural network method to evaluate the product modeling items. The mapping relationship model between morphological feature space and imagery cognitive space was constructed based on multiple linear regression equations, and the multiple regression model for each affective dimension was ideal. The results show that the model performance is reliable. The weights are calculated, and the appropriate people are selected to score and calculate the modeling scheme, and finally, the satisfactory product modeling scheme is obtained.

## 1. Introduction

Along with the progress of social history and the continuous improvement of human industrial civilization, people's living standards and consumption concepts have also undergone great changes. The esteem for material functions has gradually evolved into a strong pursuit of the field of spiritual consciousness. With the intersection and integration of various disciplines, many researchers have brought genetic ideas from biology to the discipline of industrial design; with the rapid development of computer and electronic information technology, the field of computer-aided industrial design has also gradually developed, and this design trend has led to more and more advanced algorithms to control the design process, resulting in many new design models [1]. These have brought a new idea in product design, i.e., how to assist in the design and optimization of product shape with the help of computers to produce products that are competitive in the market. Therefore, this thesis is based on a multilayer perceptron genetic algorithm neural network based on a computer-aided designer to design and optimize the product shape and find more possibilities and innovations to make the designed product more unique and selling point.

Neural networks are a research hotspot in the field of machine learning. Artificial neural networks have features such as massively parallel processing, distributed information storage, and good self-organization and self-learning ability. Artificial neural networks have been successfully applied to many fields such as signal processing, pattern recognition, and intelligent control [2]. At the same time, neural network learning also suffers from the disadvantages of easily falling into local minima, slow convergence of network learning, and complex network topology design, which hinder its application. A multilayer perceptron neural network is a forward-structured artificial neural network also called a multilayer feedforward network, that maps a set of input variables to a set of output variables and gives a prediction of the outcome of the output variables as well as a prediction model based on the input variables. Structural characteristics of multilayer feedforward networks: (1) There is no connection between neurons in the same layer. (2) There is full connectivity between neurons in two adjacent layers. (3) There is directionality in information transfer. The feedforward computation is performed layer by layer from the input to the output. The idea of a genetic algorithm is derived from the biological evolutionary process in nature and is an optimization algorithm for solving complex problems. Intelligence and essential parallelism are the biggest differences between evolutionary computation and traditional optimization methods. Evolutionary computation does not require the objective function of the object to be continuous and differentiable, and these advantages it has made it more suitable for solving complex optimization problems, and it can also be used to avoid various defects of traditional neural networks themselves [3]. By combining the multilayer perceptron neural network algorithm with a genetic algorithm, different features are obtained by different feature extraction methods for the characteristics of product modeling design, and then the genetic optimization algorithm is used to optimize the selection of the extracted features, and the classifier is trained by MLP, and the results show that the combined model achieves the expected classification effect with a high accuracy rate. Nowadays, with the development of electronic information technology, the methods for signal processing are even more endless and become more and more efficient, and people will be more thorough in the study of feature signals to make new contributions to the future development of product modeling design [4].

## 2. Status of Research

There is a lack of information on the direction of machine learning algorithms combined with product form design. Many scholars and experts in the research of product morphology design theory and machine learning have made great contributions to these fields. Literature [5] first proposed a morphological analysis method, which encodes the main morphological elements and components of a product and forms different morphological products by arranging and combining them. This approach aims to generate new design solutions through “reconfiguration” and has since been widely used in product form design and related fields. Form quantization, proposed in [6], is characterized by the concept of averaging and complementing a set of similar product forms with low correlation, extracting representative forms, giving them different weights in the process, and then deriving new forms. In terms of morphological expansion, literature [7] considers the shape as a finite arrangement of lines and sets some conditions on the shape, such as position, size, and direction, through the concept of Euclidean transformation, to generate new shapes. The imagery diagram method proposed by [8] suggested that the pictures and information can be studied by classifying them according to certain rules to establish the target scenario as a way to help the designer in designing. However, this method can only help designers to organize their thoughts to promote the association and is only an auxiliary technique before designing. Literature [9] proposes a product form design method based on the user's behavioral imagery capabilities, compared to traditional research methods that do not integrate user experience into product form design, through the study which found that the experience brought to the user by the product form has an impact on the consumer's purchase process and even plays a decisive role in the purchase decision. Literature [10] constructed a user semantic driven approach for product form prototyping and argued that semantics is the chain between people and things, and through the analysis of user semantics, it can improve user satisfaction with the product and promote the iteration of enterprise products. In addition, literature [11] proposed a theory of pan-community product form design approach based on shape literature and integrating anthropological and psychological theories. This theory first analyzes the product form elements and divides the homogeneous products and heterogeneous products and then deduces the shape grammar for both the homogeneous products and heterogeneous products and filters them to get a satisfactory solution. Literature [12] proposed a discrete neural network model with fully interconnected network topology and successfully solved the traveler problem using energy function. Literature [13] proposed a continuous neural network model, stating that neurons can be implemented with operational amplifiers and stating that the connections of all neurons can be simulated with electronic circuits, called continuous Hopfield networks. Literature [14] provides an exhaustive analysis of the error backpropagation algorithm for multilayer feedforward networks with nonlinear continuous transfer functions, which is known as the BP algorithm. Literature [15] simulates the consumer's imagery evaluation pattern for product color matching based on BP networks and generates offspring to optimize the color matching design by genetic algorithm to speed up the design process. Literature [16] incorporated genetic and biological coding methods into product color scheme design, proposed to form codes in terms of product formation, and created a PCIDBMT prototype system based on the above theory; based on interactive genetic algorithm, in [16] Yuan and Moayedi used techniques such as color merging and primary color extraction to establish an automatic mapping mechanism of color schemes from flat images to three-dimensional models of products; literature [17] introduced color matching case and grayscale correlation analysis into color matching design and used a scissor lift as an example to demonstrate that the described method can realize the conversion between case color matching and target color matching. Literature [18] proposes an orthogonal-interactive genetic algorithm, which reduces the genetic race space by orthogonal analysis to increase the convergence speed while reducing the psychological burden of fatigue to the user by reducing the number of user interactions, producing a higher adaptation value that meets the needs of product styling design.

## 3. Product Styling Design Evaluation Method Based on Multilayer Perceptron Genetic Algorithm Neural Network Algorithm

### 3.1. Principle of Multilayer Perceptron Based Genetic Algorithm Neural Network Algorithm

A perceptron is a neural network with a single layer of computational units, which is a feedforward network with no connection between neurons within the same layer and no feedback between neurons between different layers, and the signal is transmitted from the lower-layer neurons to the upper-layer neurons. Its input and output are discrete values, and the neuron determines its output by a threshold function after the weighted summation of the inputs. The perceptron is a simple nonlinear neural network with a threshold function added to the linear neurons, also known as linear threshold elements. It can accept real type signals while outputting binary discrete quantities (0, 1). The main feature of the multilayer perceptron genetic algorithm neural network is to calculate the adaptation value based on the user's interaction evaluation rather than a function formula. Because of the combination of user evaluations as well as specific function formulas, it excels in problems where it is difficult to build adaptation functions, such as in the fields of product design, image retrieval, and design evaluation. The single-layer perceptron model has only two layers of neurons, the input and output layers, which are directly connected. It is designed as follows: first step: initialize the connection rights and thresholds; the initial values of both are generally set to smaller nonzero random numbers. Step 2: The input signals are fed into the network, the connection weights of all the input signals are weighted and processed, and the result of the calculation is used as the actual output of the network. Step 3: Adjust the weights. If the actual output of the network differs significantly from the desired output, the connection weights parameter is adjusted, and the adjustment process relies on the perceptron learning algorithm automatically [19]. Step 4: Perform step 3 repeatedly until the difference between the actual and desired outputs of the network meets the predesigned requirements.

In a neural network, perceptrons can be viewed as individual nodes in the neural network. The design idea of a parameter learning scheme for a multilayer perceptron network is that, in a multilayer perceptron network, the weights of all neurons except the last neuron are set in advance, and then the perceptron learning algorithm is used to learn the weights of the last neuron. Because the weights of the first layer neurons are set artificially, the degree of excellence of the first layer neuron design will directly affect the performance of the multilayer perceptron model. The design of the first layer neuron depends on the level of understanding of the problem faced and the data, which leads to the fact that there is no general approach to the design of parameters for the first layer neural network in solving a variety of different problems. As can be seen from Figure 1, the structural characteristics of multilayer feedforward networks are (1) no connections between neurons in the same layer, (2) Full connectivity between neurons in two adjacent layers, and (3) there is directionality in information transfer. The forward calculation is done layer by layer from the input to the output [20].

The genetic algorithm improved multilayer perceptron neural network model is essentially the application of the genetic algorithm to extensively search the solution space of the target information, followed by locating the better multilayer perceptron neural network form searched by the genetic algorithm and then by training to obtain the optimal result of the prediction problem. Artificial neural networks are characterized by massively parallel processing, distributed information storage, and good self-organizing and self-learning capabilities. The process of genetic algorithm optimized multilayer perceptron neural network includes three parts: determining the multilayer perceptron neural network connection structure, determining the genetic algorithm optimized multilayer perceptron neural network weights and thresholds, and multilayer perceptron genetic algorithm neural network model prediction, the main steps are as follows (Figure 2): (1) determine the multilayer perceptron neural network structure based on the training sample data; (2) BP neural network hidden layers and layers are determined; (3) the length of the individual coding of the genetic algorithm is determined, and this value is determined by combining the number of parameters of the multilayer perceptron neural network; (4) the fitness value is optimized, and this value is optimized according to the error obtained from the training of the multilayer perceptron neural network; (5) the optimal solution is determined by the cyclic operation (4); (6) the optimal threshold weights are redetermined even more for the optimal solution; (7) the optimal weights and thresholds are assigned to the multilayer perceptron neural network model; (8) error calculation judgments on the new weights and thresholds are done to carry out multilayer perceptron neural network model training prediction; and (9) prediction result analysis is done, comparing the prediction results of multilayer perceptron neural network and genetic algorithm neural network.

Thresholds and weights of the multiperceptron neural network are cascaded according to a specific order, and the weights and thresholds of the multiperceptron neural network are cascaded according to the order; namely, N chromosomes are generated randomly; implicit and output layer thresholds; input and implicit layer thresholds; implicit and output layer weights; input and implicit layer weights; the fitness function selects the mean square error, and the fitness of the chromosomes is recalculated according to the mean square error function to judge whether the prediction results meet the target requirements and generate new individuals if they do not meet the requirements; the specific operation is to perform variation operation, crossover operation, and replication operation on the individuals that meet the requirements of the fitness value and judge whether the new individuals meet the requirements of the mean square error value function if they meet the requirements [21]. There are four mutation operations in the evolution of a multilayer perceptron genetic algorithm neural network: adding connections, adding nodes, correcting connection weights, and changing the excitation function response. If the requirement is not met, the fitness of the chromosome is calculated again according to the mean square error function, and if the requirement is met, the optimal individuals are sequentially split and the threshold and weights applied to the multisensors neural network are updated; then the multisensors neural network is forward propagated, the global error is calculated, the weights and thresholds of the network parameters are adjusted and corrected, and the multisensors neural network learning training is cycled until the set learning times or accuracy requirements, the calculation is terminated, and the results are output.

Let the input layer of a multilayer perceptron genetic algorithm neural network have *n* one input neuron, the layer has *m* one output neuron, the hidden layer has *q* one hidden layer neuron, the connection weight between the hidden layer and the output layer is *w*_*ik*_ the *v*_*ik*_ connection weight between the input layer and the hidden layer is *f*_2_, the transfer function of the hidden layer is *f*_1_, and then the output of the hidden layer neuron is calculated as follows:

(1) $$\begin{array}{c} E\left(w_{ik}\right)=n\times f_{1}\left(q\right)\times f_{2}^{m}\left(v_{ik}\right)+C_{v}. \end{array}$$

The output of the output layer neurons is calculated as follows:

(2) $$\begin{array}{c} \varphi_{0}=F\left(f^{P}\left(i\right),f^{Q}{\left(j+1\right)}^{2}\right). \end{array}$$

At this point, the multisensors genetic algorithm neural network completes the forward propagation process and establishes the mapping *n* from dimensional space vector to *m* dimensional space. For all the training samples in the BP neural network, the global error of the network is noted as *G* and is calculated as follows:

(3) $$\begin{array}{c} G=f^{P}\left(i\right)\;⊕f^{Q}\left(j\right)=f\left(P_{i}\right)f^{Q}{\left(j\right)}^{T}. \end{array}$$

The variation in the output layer weights of the multisensory layer genetic algorithm neural network is noted as *L* and is calculated as follows:

(4) $$\begin{array}{c} L=\sum_{\left(i,j,k\right)\in D}-\ln\;\sigma \left(z_{ij}-z_{ik}\right). \end{array}$$

The formula for adjusting the weights of each neuron in the output layer is obtained as

(5) $$\begin{array}{c} R_{n+1}=R_{n}^{2}-\sum P_{ij}. \end{array}$$

Fixed topology evolution must be done artificially to design the topology of the neural network. In contrast, topological weight evolution methods can automatically evolve the correct network topology. In addition, there is no general set of laws that guarantee excellent performance of artificially designed neural networks, so the topology of multisensory neural networks evolved based on genetic algorithms tends to outperform artificially designed solutions in terms of performance. This phenomenon is particularly evident in keeping network complexity to a minimum [22]. Although topology weight evolution methods perform better compared to fixed topology evolution methods, they also face many problems that do not exist in fixed topology evolution methods. There are four mutation operations in the evolution of a multilayer perceptron genetic algorithm neural network: adding connections, adding nodes, correcting connection weights, and changing the excitation function response. Before the mutation operation, we set a mutation probability, and the mutation of connection weights is done by correcting all connection weights according to the set mutation probability. In special cases, it is also possible to disregard the mutation probability and directly turn the original weight into a new weight. The mutation is used to change the weights and the network structure. Mutation of connection weights is done by adding a floating-point number (either positive or negative) to each weight with a fixed probability that matches a normal distribution. The network structure is mutated in two ways: mutation by adding nodes and mutation by adding a connection between two nodes.

### 3.2. Product Styling Design Evaluation Methods Based on Machine Learning Algorithms

The so-called modeling is to point, line, surface as the basic elements, according to certain rules of mutual transformation, organic to produce new organic form. In the process of styling, the use of more organic forms of free-form products can increase the uniqueness and innovation of products, of which, “selection” and “change,” as two major modeling laws, are often applied. The so-called selection is to choose the basic type according to the use of function, maneuverability, and other conditions. There are two types of basic shapes, geometric and organic. Geometric forms are some common geometric shapes in mathematics, while organic forms are streamlined, bionic, or free-form. Transformation is the operation of dividing, cutting, accumulating, merging, stretching, extruding, bending, etc., in the form of the basic type. Splitting: It is in the form of “loss” or “separation.” Usually, when cutting, it will be divided according to the golden ratio; for example, we commonly see the ratio of wheelbase to the total length of cars and the ratio of screen to the key distribution of flat panel products, etc., which are all golden ratios. Cutting: The basic type is partially cut to produce a face change in shape. The idea of the genetic algorithm comes from the biological evolution process in nature and is an optimization algorithm for solving complex problems. Intelligence and essential parallelism are the biggest differences between evolutionary computing and traditional optimization methods. The position, curvature, and depth of the cut all make the product produce different new shapes. Accumulation: The same or similar monoliths are stacked in size, position, number, and direction to produce a regular stack. The fruit plate, for example, is a shape produced by the accumulation of a basic type. (4) Merging: It is taking two separate individuals and creating a new shape by intersecting, cutting, or superimposing them. This type of shape can usually be seen in mechanical parts. (5) Stretching: As the name suggests, this is taking a base shape and dragging it outward in a given direction to produce a new shape. This type of molding is seen everywhere in life; for example, refrigerator and cabinet air conditioner molding are applications of this method. (6) Extrusion: On the surface of a monolith, stretching in the direction of centripetal force is called extrusion.

With the vigorous development of computer technology, parametric and quantitative technology has become a hot spot for research in various academic fields and is also gradually applied to product form design. Most of the product form design is an improved design based on the original shape, and its parameters have a clear correspondence with the size of the design object. Therefore, the parametric design brings a more efficient design process to product design, which can use the previously accumulated and established models and modify them on this basis. The principle of parametric design is that the parameters of a line or a figure correspond to the control dimensions of the design object, and when different values of the parameter sequence are given, the design result changes, i.e., a new geometry is obtained under the drive of the parameters. At present, the application of parametric design in morphological design is more extensive, and its scope is gradually extended to the whole life cycle of the product, including two-dimensional organization, three-dimensional entities, accessories intermediate relations, product features expression, and other product-level designs.

Product styling is a process of multiple solution selection, and at the same time, styling is a field full of emotions. If traditional machine learning algorithms are involved in the design process, the nonoptimal individuals are completely discarded while the good individuals are retained. However, in the design domain, nonoptimal individuals can still have some influence and contribution to the final solution product even if they fail to satisfy some specific requirements. Therefore, this requires the introduction of multilayer perceptron neural networks to control the genetic algorithm. The main feature of the multilayer perceptron genetic algorithm neural network is to calculate the adaptation value based on the user's interaction evaluation rather than a function formula. Since users' visual cognition of products is mainly reflected in the form of perceptual information, designers should take the initiative to obtain information about users' perceptual preferences and understand how users decode their cognition of products and their perceptual preferences, to ensure success of design coding. Because of the combination of user evaluations as well as specific function formulas, it excels in problems where it is difficult to build adaptation functions, such as in the areas of product design, image retrieval, and design evaluation. For example, Figure 3 shows the flow chart of the product interactive styling design model.

In the conceptual stage of product design, the principle of combinatorial innovation is often used to generate new shapes. Combinatorial innovation, as it means, is the process of segmenting and analyzing a product based on a certain aspect, so that the modules can be combined to produce a new product shape, based on, but not limited to, function, shape, structure, man-machine, material, etc. The process of design is always accompanied by many uncertainties, how to translate the subjective design activities into the digital language to analyze and quantify the emotions and demand preferences, need to analyze, process, and integrate all kinds of complex elements with the help of scientific and effective evaluation methods. Hierarchical analysis (AHP) is commonly used to measure the emotional factors of a product, simplifying complex decisions, or apply the principles of perceptual engineering theory to establish and determine the final evaluation index through semantic difference hierarchical evaluation. Product design evaluation is to use specific rules to evaluate the attribute values of each solution in a limited set of solutions and then use the specific rules to obtain a comprehensive evaluation value and finally rank all solutions based on the comprehensive evaluation value and obtain the optimal solution. It generally includes three steps: (1) normalize the evaluation matrix; (2) determine the weight size of each solution; (3) rank all alternatives. Commonly used design evaluation methods include the simple linear weighting method, efficacy coefficient method, hierarchical analysis method, approximate ideal solution ranking method, gray correlation analysis method, etc. The simple linear weighting method is a common multiobjective evaluation method; this method is based on the actual situation; first, determine the evaluation attribute weights, and then standardize the decision matrix, find out the average value of the linear weighting index of each option, and use it as the judgment basis of each feasible option ranking. The efficacy coefficient method converts the dissimilarity measures of each attribute into corresponding dimensionless efficacy coefficients and then performs a comprehensive evaluation. TOPSIS is a ranking method that approximates the ideal solution, which is characterized by full utilization of the original data, low error, and high reliability. The optimal solution is the one closest to the positive ideal solution and farthest from the negative ideal solution, to evaluate the optimal solution. The gray correlation method is a multifactor statistical analysis method, which is based on the sample data of each factor and analyzes the correlation size between each component factor and the whole and reflects the similarity of the solution to be evaluated and the optimal solution in terms of shape. Based on the multilayer perceptron genetic algorithm neural network, these evaluation indexes can be connected in series to evaluate the product shape design in a multifaceted way.

## 4. Experimental Verification and Conclusions

To verify the feasibility and effectiveness of the proposed method, a series of experiments are conducted to illustrate this paper. The main steps include the following: (1) constructing an evaluation system using perceptual engineering and hierarchical analysis; (2) using hierarchical analysis to obtain subjective weights; (3) using entropy weighting to obtain objective weights; (4) using game theory to obtain comprehensive weights; (5) using SD method to build a perceptual decision matrix; and (6) using KE-GRA-TOPSIS method to rank the alternative products.

A comprehensive evaluation system for the product was developed using perceptual engineering and hierarchical analysis. The target level has only one element, i.e., the selection of the product solution. Six criteria and 12 indicators were identified based on the TF-EPA method. The product perceptiveness was evaluated in 6 dimensions: gender perspective, acceptance, structural characteristics, duration, weight characteristics, and technical characteristics, respectively. Two indicators were included under each criterion and the indicators consisted of a pair of perceptual words.

The relative closeness trends of the three methods MLP, GA, and GA-MLP-NN regarding the 14 alternatives were obtained based on the experiments, and the comparison graphs shown in Figure 4 were drawn. In the GA method, the relative closeness gap of the alternatives is larger because the GA method only considers the distance of the alternatives in space and magnifies the evaluation results; the gap of the alternatives in the MLP method is smaller because the method focuses on the association between indicators but ignores the distance of the evaluation alternatives in space. Introduce the preference information in the user's multidimensional perceptual preference space directly into the design conception. The information transfer and transformation efficiency in the process is improved. The GA-MLP-NN method is an integration of the GA method and MLP, which considers the relative closeness derived from this method is more realistic as it considers both the degree of association between evaluation options and the gaps between options.

The results of DM selection were also compared with those of the MLP method, GA method, GA-MLP-NN method, and TOPSIS method, and the comparison results are shown in Figure 5. The KE-GRA method was not included in this comparison test because its accuracy was too low. The GA-MLP-NN method had an accuracy of 78.6%, followed by the MLP method with 57.2%. Also, the accuracy of the GA method and TOPSIS method was 7.2% and 0. Observing Figure 5, it can be seen that the results of the GA-MLP-NN method and MLP method were similar, while the GA method and TOPSIS method were similar. In addition, the results of the GA-MLP-NN method and the MLP method are roughly consistent with the choice of DM. This experiment verifies that the TOPSIS method and its extensions cannot be directly used for the perceptual ranking of products.

To verify the validity of the proposed method, 10 additional participants were invited to repeat the experiment.  Figure 6 shows the results of preferences and alternatives ranking given by the participants. It is worth noting that the subjective weights in the hierarchical analysis method are adjustable. The comparison results of the subjective choice results of the 10 participants with the GA-MLP-NN method and the MLP method are shown in Figure 6, which contains the comparison of the number of correct rankings and the comparison of the accuracy rate. In this case, the bar graph represents the number of correct rankings and the line graph represents the accuracy rate. In the GA-MLP-NN method, the accuracy rates of U1 to U10 are 85.7%, 100%, 85.7%, 100%, 100%, 100%, 85.7%, 100%, 100%, 100%, and 100%, in that order. The average accuracy was calculated to be 95.7%. In the MLP method, the accuracy rates of U1 to U10 were 85.7%, 85.7%, 85.7%, 85.7%, 85.7%, 85.7%, 85.7%, 71.4%, 85.7%, 100%, and 85.7% in that order. The average accuracy rate was calculated to be 85.7%. In terms of accuracy, both the GA-MLP-NN method and the MLP method performed well, and the GA-MLP-NN method was more accurate. The above results show the feasibility of the perceptual decision matrix and that the proposed GA-MLP-NN method can accurately rank products according to users' personalized preferences.

In Figure 7, True Positive (TP) indicates the number of positive samples classified as positive; True Negative (TN) indicates the number of negative samples classified as negative; False Positive (FP) indicates the number of negative samples classified as positive, and False Negative (FN) indicates the number of positive samples classified as negative. The commonly used evaluation metrics, including Accuracy, Precision, Recall, False Discovery Rate (FDR), and False Positive Rate (FPR), are listed in Figure 7. 30 product images are arbitrarily selected as a content map and 10 images as style map; 300 new product images were generated. After mixing 100 real images and 300 generated images, the 30 users in Section 3.4.2 were invited to distinguish the truth from the falsehood of 400 images. Since the product images generated by the GA-MLP-NN method are only used to inspire designers or users and are not final design renderings, to weaken the detailed features of the generated images, 30 users (with normal vision) observe the images at a distance of 1 m from the display (resolution of 2560 × 1440) with a maximum display size of about 8 cm on one side (width or height) of the images and each image. The dwell time does not exceed 2 s. The purpose of this experiment is to evaluate the user's ability to distinguish between real and generated images and to reflect the quality of the generated images. FDR is the proportion of actual negative samples among positive samples, and FPR is the proportion of actual negative samples among positive samples. FDR and FPR are positive indicators. The calculated FDR and FPR are 69% and 67%, respectively, indicating that the generated images are of good quality and can be used to display and inspire designers.

Due to the relationships of relevance, subordination, redundancy, and similarity between adjectives, two perceptual words with similar concepts and opposite meanings are more reflective of user psychology. Therefore, perceptual words are selected in this chapter to describe the user's psychological feelings. The importance of a word is proportional to the number of times it appears in a text, and if a word appears repeatedly in the text under study, it can be used to characterize the dominant tendency of the text. Considering the one-sidedness of the traditional method of selecting sentiment words by considering only word frequency or user preference in sentiment engineering, this chapter proposes a GA-MLP-NN-based method for selecting sentiment word pairs based on the characteristics of word frequency and EPA dimensions. Text sentiment analysis is the use of computer analysis of text with subjective feelings in user comments for polarity classification, which is usually classified as positive (positive), derogatory (negative), or neutral. Sentiment classification methods can be divided into two categories: machine learning-based methods and lexicon-based methods, the latter of which discriminate text sentiment by sentiment lexicons such as WordNet and HowNet, which rely on the quality and continuous improvement of sentiment lexicons. In this chapter, the sentiment dictionary-based approach is used to determine the sentiment tendency of sentiment words in online reviews. The HowNet dictionary and synonym word forests are searched to obtain the results of sentiment tendency judgment of sentiment words. The score of sentiment unit EO is the product of sentiment polarity EP and sentiment intensity EI, and the sentiment evaluation of the whole text is characterized by aggregating the sentiment units in the text. The sum of the sentiment tendency scores of independent positive and negative sentiment words in a sentiment pair is used as the evaluation value of a set of sentiment word pairs. Commonly used design evaluation methods include the simple linear weighting method, efficacy coefficient method, hierarchical analysis method, approximate ideal solution ranking method, gray correlation analysis method, etc. The perceptual evaluation values of the six sets of perceptual words are obtained by traversing the product reviews according to the perceptual evaluation value calculation process, where positive values indicate that the sample ratings are biased towards positive perceptual words, negative values indicate that the sample ratings are biased towards negative perceptual words, and the absolute values of the ratings indicate the degree of deviation. In the perceptual evaluation of the sample in Figure 8, the perceptual word “good-poor” is rated as 0.949, indicating the overall product evaluation preference; “beautiful-ugly” is rated as 2.133, indicating the product. The “smooth—sluggish” rating of −1.005 indicates that the system is sluggish to use. The perceptual rating for sample 2 was medium, with a “large-small” rating of 1.957, indicating a large product size. The perceptual rating for sample 3 was medium, with a “large-small” rating of 2.127, indicating a large product size. Sample 4 had a medium perceptual rating of 4.0 on the “large-small” scale, indicating a large size, and a −1.121 on the “easy-fussy” scale, indicating that the product was fussy to use. The “Smooth-Sluggish” rating of 3.0 indicates that the system is smooth to use. The perceptual rating for sample 5 was medium, with a rating of 2.5 for “beautiful-ugly” indicating a beautiful product, and 2.589 for “large-small” indicating a large product size. The “Flow-Sluggish” rating is 0.953, which indicates smooth system usage. The model predicted by GA-MLP-NN and the actual value model almost agree, indicating that the GA-MLP-NN model has high accuracy.

With the widespread application of the Internet of Things, Internet, and automation technologies, products are developing in the direction of intelligence and information technology, and the whole product life cycle process is becoming more and more open and transparent. The product life cycle is the whole process from product development to end-of-life, including product design, production and processing, transportation and supply, and sales and use. The data generated from the whole product lifecycle includes data in the database of enterprise information management system such as enterprise resource planning, CRM, manufacturing enterprise production process execution system, product data management, and supply chain management, as well as data generated by users in the Internet and e-commerce system such as browsing, clicking, purchasing, and reviewing, etc. These data have the typical characteristics of big data, i.e., many data types, large data volume, low-value density, and high commercial value. These data have the typical characteristics of big data, namely, many data types, large data volume, low-value density, and high commercial value. Among them, the data types include text data, image data, voice data, video data, and log data. These product-related data grow exponentially every day to form the product life cycle big data. The multilayer perceptual genetic algorithm neural network based on this paper can make full use of the characteristics of big data with low-value density and high commercial value to extract valuable information from large-scale data and the value of the most core part. The value of big data depends on the role that the data analysis results play in the application. The field of product design has received slightly less attention than other applications of big data, but there is no shortage of roles it can play. For example, by collecting product reviews in e-commerce systems, it is possible not only to detect changes in user needs but also to improve product defects based on user feedback, thereby increasing user satisfaction. Image big data can intuitively inspire designers and facilitate product styling.

## 5. Conclusion

This paper further develops an intelligent and systematic approach to product innovation design by exploring how to obtain information related to product design from the big data generated from the product life cycle and analyzing it in depth using techniques such as genetic algorithm neural network model based on multilayer perceptron, and the main research work is as follows. This paper analyzes the advantages and disadvantages of each multilayer perceptron neural network as well as genetic algorithm, and by combining genetic algorithm with multilayer perceptron neural network model, a set of multilayer perceptron genetic algorithm neural network models is formed, and product design domain knowledge is incorporated into it, and the method can automatically identify, extract, and reconstruct the content and color features of images and migrate them to the product shape in the content map. Real-time generation of new product images is achieved. Among them, the training of the multilayer perceptron neural network migration model is an unsupervised training based on image data, and the trained model is used to automatically migrate the stylistic features of stylistic images; the genetic algorithm model is a supervised training, and the trained model is used to predict the product semantics in the content graph and guide the selection of the stylistic graph. The method alleviates the problems of poor image quality, uncontrollable content, and lack of theoretical guidance in the product design domain of the generated solution. The subjective imagery of users is ambiguous, and there is a “black box” problem between their subjective evaluation value and the elements of product form and shape. It is also not easy to improve the competitive advantage of the product. This paper also integrates product design domain knowledge into textual big data techniques to propose a data-driven perceptual engineering approach for online reviews. In terms of perceptual word collection, online reviews are used as a source of perceptual words; in terms of perceptual word acquisition, a GA-MLP-NN perceptual word extraction method combining three dimensions of word frequency and EPA is proposed; in terms of perceptual evaluation, a perceptual evaluation value calculation method combining degree adverbs with word clustering for online reviews is proposed, and the basic idea is to obtain users' emotional tendency towards the product by mining the emotional tendency of perceptual words. In terms of mapping model construction, a multilayer perceptron genetic algorithm neural network is used to construct a relationship model between users' difficult-to-quantify perceptual needs and product design elements, while the models constructed by multiple linear regression methods are compared to verify the effectiveness and feasibility of the proposed method.

## Figures and Tables

**Figure 1:** Topology of multilayer perceptron neural network.

**Figure 2:** Computational flow of neural network of multilayer perceptron genetic algorithm.

**Figure 3:** Flowchart of an interactive product styling model.

**Figure 4:** Comparison of relative posting progress trends.

**Figure 5:** Results of comparison of program ranking.

**Figure 6:** Results of participant preferences.

**Figure 7:** Partial sample attribute parameter rank distribution.

**Figure 8:** Partial sample perceptual evaluation.

## Data Availability

The data used to support the findings of this study are available from the corresponding author upon request.
